# Blood Vessel Segmentation of Fundus Retinal Images Based on Improved Frangi and Mathematical Morphology

**DOI:** 10.1155/2021/4761517

**Published:** 2021-05-26

**Authors:** Feng Tian, Ying Li, Jing Wang, Wei Chen

**Affiliations:** College of Communication and Information Engineering, Xi'an University of Science and Technology, Xi'an 710054, China

## Abstract

An improved blood vessel segmentation algorithm on the basis of traditional Frangi filtering and the mathematical morphological method was proposed to solve the low accuracy of automatic blood vessel segmentation of fundus retinal images and high complexity of algorithms. First, a global enhanced image was generated by using the contrast-limited adaptive histogram equalization algorithm of the retinal image. An improved Frangi Hessian model was constructed by introducing the scale equivalence factor and eigenvector direction angle of the Hessian matrix into the traditional Frangi filtering algorithm to enhance blood vessels of the global enhanced image. Next, noise interferences surrounding small blood vessels were eliminated through the improved mathematical morphological method. Then, blood vessels were segmented using the Otsu threshold method. The improved algorithm was tested by the public DRIVE and STARE data sets. According to the test results, the average segmentation accuracy, sensitivity, and specificity of retinal images in DRIVE and STARE are 95.54%, 69.42%, and 98.02% and 94.92%, 70.19%, and 97.71%, respectively. The improved algorithm achieved high average segmentation accuracy and low complexity while promising segmentation sensitivity. This improved algorithm can segment retinal vessels more accurately than other algorithms.

## 1. Introduction

Blood vessel segmentation of fundus retinal images can help doctors in diagnosing multiple eye diseases. Segmenting blood vessels integrally and accurately is necessary for accurate analysis of main blood vessels and branches [1]. Currently, physicians mark blood vessels manually according to experiences, which is characterized by low efficiency and easy interference by subjective factors [2, 3]. Therefore, the automatic segmentation of retinal vessels is of important significance [4, 5].

Gray distribution of fundus retinal images is uneven due to influences of noises, artifacts, and illuminations, accompanied by low contrast between blood vessels and background. Moreover, arteries and veins in images cross over and superpose mutually, thereby resulting in difficulties of segmentation. The existing blood vessel segmentation methods of fundus retinal images include supervised and unsupervised learning. The former requires training according to the provided standard training set and uses the trained classifier to segment blood vessels in unknown images. The latter requires no training but segments blood vessels through thresholding the filtering response or depending on methods on the basis of certain rules.

Without artificial prior marking information, the retinal vessel segmentation method on the basis of unsupervised learning has a small workload and high working efficiency. Currently, unsupervised segmentation methods include methods on the basis of windows [6–13], vessel tracking [14–20], and morphological operations [21–23].

Chaudhuri et al. [6] were the first to propose blood vessel segmentation by using the Gaussian filter. Subsequently, Li et al. [7] proposed a segmentation technique by combining a multiscale matched filter and dual-threshold method. Kaur and Sinha [8] proposed a segmentation algorithm on the basis of Gabor filter and gray cooccurrence matrix. Wang et al. [9] processed the coarse and fine blood vessels by using the multiscale 2D Gabor wavelet. Singh and Srivastava [10] proposed a method on the basis of the extended matched filter. Cruz-Aceves et al. [11] segmented blood vessels by using a multiscale Gabor filter and threshold segmentation method on the basis of multiobjective optimization. Aguirre-Ramos et al. [12] enhanced the blood vessel structure and its profile by using the Gabor filter and Gaussian distribution derivatives. Singh and Srivastava [13] proposed a matched filtering technique centered at the Gumbel probability distribution function to improve retinal vessel segmentation performances. These methods, which are based on windows, can maintain the original vessel structure but require the processing of each pixel, thus leading to heavy computational workloads and long segmentation time.

Frangi et al. [14] introduced the Hessian matrix into the extraction of characteristic directions of images. Kumar et al. [15] extracted blood vessels from retinal images on the basis of inherent characteristics of LoG and MF, which avoided misclassification of nonvascular pixels. Fathi and Naghsh-Nilchi [16] proposed a multiscale vessel segmentation algorithm based on continuous wavelet transform. Qian Zhao et al. [17] put forward an algorithm on the basis of level set and regional growth. Rezaee et al. [18] proposed an optimized segmentation technique of retinal vessels that combined adaptive filtering, fuzzy entropy, and skeletonization. Ghoshal et al. [19] proposed a method to enhance fine blood vessels by vascular area and axial ratio. Zhao et al. [20] developed an infinite activity profile model for retinal vessel segmentation through the information of the image hybrid region. These methods on the basis of vessel tracking can acquire local features of blood vessels. However, they cannot realize continuous tracking due to branches or intersections, resulting in poor segmentation accuracy.

Rodrigues and Marengoni [21] proposed an optic disc detection algorithm on the basis of wavelet transform and mathematical morphology. The proposed algorithm segmented veins and arteries in retinal images according to tubular characteristics of blood vessels. Rodrigues and Bezerra [22] applied morphology and topology extractor to extract pixels of the vascular tree and discovered topological vascular characteristics and connectivity. Neto et al. [23] proposed a coarse-to-fine vascular detection method of retinal images. First, this method implemented general vessel segmentation. Second, refined vessel segmentation was performed on the basis of curvature analysis and morphological reconstruction. These methods on the basis of morphology are fast, highly efficient, and satisfactorily inhibit noise. However, they rely highly on the selection of structural elements.

In this study, a vessel segmentation method of fundus retinal images on the basis of the improved Frangi and mathematical morphology was proposed by combining vessel tracking and morphological operation. First, the fundus retinal image was preprocessed by global enhancement. Second, blood vessels were enhanced by the improved Frangi filtering method. Third, noise interferences surrounding the fine blood vessels were eliminated by the improved mathematical morphological method. Last, vessel segmentation of the retinal image was performed through the Otsu threshold segmentation method.

## 2. Vessel Segmentation of Retinal Images

### 2.1. Image Preprocessing

Fundus retinal images are in RGB format, which generally have to be transformed to single-channel images for the convenience of computer processing. Images in R, G, and B channels were compared (Figure 1). Blood vessels in the G channel image have high contrast with the background. Therefore, the G channel image was chosen for preprocessing.

Enhancement of fundus retinal images can distinguish blood vessels from other background regions. Histogram equalization processing can enhance the contrast of each object in a specific image, in which the scope of image intensity will be extended. As fundus retinal images have low contrast and the vascular region is dark with low contrast, the global histogram equalization method fails to achieve the ideal enhancement of blood vessels (Figure 2(a)).

Adaptive histogram equalization (AHE) implements histogram enhancement on each pixel by calculating the transformation function of each pixel neighbor domain. AHE is more appropriate to the local contrast of images and enhanced image edges to gain additional details. For retinal vascular images, AHE may amplify noises surrounding fine blood vessels in images while enhancing the contrast. Therefore, using contrast-limited adaptive histogram equalization (CLAHE) algorithm is essential to enhance retinal vessels because it can inhibit noise enhancement. Moreover, the CLAHE algorithm has a simple calculation and determines only one parameter of the amplitude limit.  Figure 2(b) shows the processing result of the CLAHE algorithm.

The enhancement results of Figure 2 were compared. The AHE algorithm increased the noises surrounding the fine blood vessels and in the image background while enhancing blood vessels. This feature resulted in the uneven brightness distribution of the image. On the contrary, the CLAHE algorithm decreased noise interferences while enhancing the contrast between blood vessels and background effectively.

### 2.2. Improved Frangi Filter Algorithm

Blood vessels present a linear tubular structure in fundus retinal images, and the diameter range falls within a limit. From Gaussian function and original image convolution, most structures that are smaller than scale *s* in the image can be inhibited, whereas those with a width equivalent to *s* are enhanced. Therefore, vascular responses under different scales could be expressed by convolution of the original image *I*(*x*, *y*) and Gaussian kernel *G*(*x*, *y*; *s*), whose scale *s* is the radius of the vessels:

(1) $$\begin{array}{c} I_{s}\left(x,y;s\right)=I\left(x,y\right)⊗G\left(x,y;s\right), \end{array}$$

where the Gaussian function is

(2) $$\begin{array}{c} G\left(x,y;s\right)=\frac{1}{2\pi s^{2}}e-\frac{x^{2}+y^{2}}{2s^{2}}. \end{array}$$

The original Hessian matrix of a two-dimensional image *I*_*s*_(*x*, *y*; *s*) is defined as

(3) $$\begin{array}{c} H=\left(\begin{array}{cc} \partial_{xx}I_{s} & \partial_{xy}I_{s}\\ \partial_{yx}I_{s} & \partial_{yy}I_{s} \end{array}\right), \end{array}$$

where *∂*_*xx*_*I*_*s*_, *∂*_*xy*_*I*_*s*_, *∂*_*yx*_*I*_*s*_, and *∂*_*yy*_*I*_*s*_ are second-order partial derivatives of the image. Numerical values of these four parameters can be approximate to the linear convolution of the image and the scale-normalized derivative of Gaussian kernel function [24]:

(4) $$\begin{array}{c} \partial^{n}I_{s}\left(x,y;s\right)=I\left(x,y\right)⊗s^{n}\partial^{n}G\left(x,y;s\right). \end{array}$$

Therefore, the Hessian matrix of the point *p*_0_ in the image is defined as

(5) $$\begin{array}{c} H\left(p_{0},s\right)=I\left(x,y\right)⊗s^{2}*\left(\partial^{2}G\left(x,y;s\right)\right). \end{array}$$

In a two-dimensional image, the Hessian matrix is a two-dimensional positive definite matrix that has two eigenvalues and corresponding eigenvectors. When blood vessels are low-dark tubular structures relative to the background, the Hessian matrix of the pixels at blood vessels has high positive eigenvalue *λ*_1_, small eigenvalue *λ*_2_, and |*λ*_1_| ≫ ∣*λ*_2_∣. Moreover, *λ*_1_ is higher when the brightness of the pixel at the blood vessel is lower and the blood vessel diameter is larger. Therefore, an equivalence factor *d* = 2*s* was introduced into the vascular response function to normalize responses of blood vessels under different scales.

In retinal images, eigenvalues of the Hessian matrix represent curvature intensity of blood vessels, whereas eigenvectors represent the curvature direction of blood vessels. As *λ*_1_ and *λ*_2_ are two eigenvalues of the matrix and |*λ*_1_| ≫ ∣*λ*_2_∣, the eigenvector *μ*_1_ corresponding to *λ*_1_ reflects the direction of maximum curvature (perpendicular to the axial direction of the blood vessel). By contrast, that of *λ*_2_ reflects the direction of minimum curvature (axial direction of the blood vessel). Hence, another parameter of arctan(*λ*_2_/*λ*_1_) that represents the direction angle of the eigenvectors was introduced in [25–28]. Therefore, the proposed new vascular response function is

(6) $$\begin{array}{c} f\left(p_{0},s\right)=e^{-\arctan{\left(\lambda_{2}/\lambda_{1}\right)}^{2}*\left(\lambda_{1}/d\right)}. \end{array}$$

The output result under multiscale is

(7) $$\begin{array}{c} f\left(p_{0}\right)=\underset{s_{\min\leq s\leq s_{\max}}}{\max}f\left(p_{0},s\right), \end{array}$$

where *s*_min_ and *s*_max_ are the minimum and maximum radii of blood vessels in fundus retinal images, respectively.

Figure 3 depicts the blood vessel enhancement effects on the basis of the traditional and improved Frangi filter. The vascular response function on the basis of the traditional Frangi filter will strengthen noises to a large extent while enhancing blood vessels. Thus, many false-positive pixels are generated in the marginal area of field of view (FOV), which influences follow-up elimination of margins of the FOV region through masking. However, the improved Frangi filter can increase the overall performance of images significantly while enhancing blood vessels. The improved Frangi filter enhances coarse blood vessels and maintains the fine ones to the maximum extent, without influencing edges of the FOV region.

### 2.3. Otsu Segmentation Algorithm on the Basis of Improved Mathematical Morphology

#### 2.3.1. Improved Mathematical Morphology

After the fundus retinal image is enhanced by the improved Frangi filter, small branches of blood vessels are enhanced. At the same time, the noises in the background are increased. Therefore, the primary goal is to eliminate noise interferences in the background region of the image while retaining fine blood vessels as much as possible before image segmentation.

Basic operations of mathematical morphology include dilation and erosion, which are defined, respectively, as

(8) $$\begin{array}{c} I_{d}=I⊗\text{Se}, \end{array}$$

(9) $$\begin{array}{c} I_{e}=I\Theta \text{Se}, \end{array}$$

where *I* is an image for processing, Se is a structural element of morphology, and *I*_*d*_ and *I*_*e*_ are images after dilation and erosion, respectively.

Open operation in morphology refers to the erosion operation of the image by using the structural element Se and then implementing the dilation operation. Open operation can eliminate bright regions of the image that are smaller than structural elements without affecting other details. Open operation is defined as

(10) $$\begin{array}{c} I_{\text{open}}=I\circ \text{Se}=\left(I\Theta \text{Se}\right)⊕\text{Se}. \end{array}$$

The structural element in mathematical morphology is very important to image processing. The linear structure was chosen as the structural element considering that blood vessels in fundus retinal images have tubular structures. This structural element has two parameters, namely, length and angle. Traditional mathematical morphology can only use the same linear structural elements (length and angle in the structural element are fixed) to process the entire image. Blood vessels in the fundus retinal image are in network distribution and have different diameters and directions. Therefore, traditional mathematical morphological processing fails to achieve the ideal effect (Figure 4(a)). Thus, an improved mathematical morphological method was proposed [29–31].

First, the lengths of linear structural element increase from the minimum diameter (2 pixels) of blood vessels to the maximum diameter (12 pixels) for every 1 pixel. Second, the angles of the linear structural element are determined every 10° from 0° to 170° given that the direction of blood vessel sections ranges between 0° and 360° and is symmetric. In this way, open operation results of 198 templates could be gained. If the gray value of the open operation results of *k*th template at the pixel point (*i*, *j*) is *I*_open_(*i*, *j*), then the gray value of each pixel point after final morphological processing chooses the maximum of 198 operation results at the corresponding position:

(11) $$\begin{array}{c} I_{R}=\underset{k}{\max}I_{{\text{open}}_{k}}\left(i,j\right), \end{array}$$

where *I*_*R*_ is the image processed by the improved mathematical morphology.  Figure 4(c) shows the result.

Figures 4(a) and 4(c) depict the processing results of the traditional and improved mathematical morphologies, respectively. Moreover, Figures 4(b) and 4(d) show the magnifications of corresponding subregions. Traditional mathematical morphology decreases partial noises but causes serious distortion of the image, and some vascular information is lost. However, the improved mathematical morphology decreases image noises significantly and sharpens image profiles and details, without causing loss of image information. These features are beneficial for subsequent segmentation.

#### 2.3.2. Otsu Segmentation Algorithm

Otsu algorithm is a high-efficiency and simple algorithm for image binarization. According to gray characteristics of images, the Otsu algorithm divides an image into background and foreground. Then, gray histograms of the background and foreground pixels were calculated, and their variances were compared to find the optimal threshold. This threshold refers to the threshold at the maximum variance and is used to distinguish background and foreground pixels.

For an image, *t* is the segmentation threshold of the background and foreground pixels. *ω*_0_ refers to the proportion of foreground pixels in the image, and *μ*_0_ pertains to the average gray level. *ω*_1_ is the proportion of background pixels in the image, and *μ*_1_ is the average gray level.

The overall average gray level of the image is

(12) $$\begin{array}{c} \mu =\omega_{0}*\mu_{0}+\omega_{1}*\mu_{1}. \end{array}$$

The variances of foreground and background pixels are

(13) $$\begin{array}{c} g=\omega_{0}*\omega_{1}*\left(\mu_{0}-\mu_{1}\right)*\left(\mu_{0}-\mu_{1}\right). \end{array}$$

When the variance *g* is at maximum, the difference between the foreground and background also reaches the maximum. At this moment, the gray level *t* is the optimal threshold.

## 3. Experimental Results and Analysis

In this study, the proposed algorithm was tested on the test set of public fundus retinal images by the DRIVE and STARE data sets. Qualitative and quantitative contrast analyses among segmentation results of the proposed method and manual segmentation of two experts and traditional Frangi filter processing were carried out. For comparative assessment, segmentation effects of the proposed method were compared with those of new algorithms. The traditional Frangi filtering process is also performed after the CLAHE-enhanced image, and then, improved mathematical morphology operations and Otsu algorithm are used for segmentation.

### 3.1. Segmentation Effect

The manual segmentation results of the two experts are the most important indicators to assess the segmentation effect of fundus retinal images.  Figure 5 shows the comparison of the vascular segmentation results of the proposed method, the manual segmentation results of two experts, and the results of traditional Frangi filtering. These images were chosen randomly from the DRIVE data set.  Figure 5(a) illustrates the original colorful fundus retinal images. Figures 5(b) and 5(c) show the manual segmentation results of the first and second experts, respectively. Moreover, Figures 5(d) and 5(e) depict the segmentation results of the traditional Frangi filter and the proposed method, respectively.

The results of manual segmentation by experts, traditional Frangi filtering segmentation, and the proposed method segmentation of three fundus retinal images which were chosen randomly from the DRIVE data set are shown in Figure 5.  Figure 6 illustrates the 1D cross sections of the middle row of marked subarea (the framed part in the first column of images in Figure 5) in the above three segmentation results. This figure also shows that the width of blood vessels segmented by the proposed algorithm is consistent with that of the manual segmentation of experts, whereas the blood vessels segmented by the traditional Frangi filter are coarse. When using the traditional Frangi filter to enhance blood vessels, optic disk pixels are very easy to be determined as vascular pixels compared with those of Figure 5. Moreover, the traditional Frangi filter tends to coarsen veins and arteries in the center, thus generating false-positive pixels surrounding blood vessels. However, the proposed method shows a good segmentation effect of retinal vessels and assures the integrity and accuracy of vessel segmentation.

Figure 7 shows the comparison of the detailed segmentation effects of the above three methods. After the traditional Frangi filtering segmentation, many vascular pixels at ends of blood vessels are lost, and many fine blood vessels that are important to analyze retinal images are missing. Comparatively, the proposed method maintains many fine blood vessels, and the whole retinal vessels are still in good structure and connectivity.

### 3.2. Performance Analysis

For the objective evaluation of the segmentation effect of blood vessels, accuracy (Acc), sensitivity (Se), and specificity (Sp) are generally applied in quantitative assessment. Acc refers to the proportion of accurately classified pixels in total pixels of fundus retinal image. Se and Sp refer to the proportion of vascular and nonvascular pixels that are recognized accurately in the segmentation result, respectively.  Table 1 shows the calculation formulas of these three indicators.

In Table 1, TP and FP refer to vascular and background pixels that are judged as a blood vessel in the segmentation result, respectively. FN and TN refer to vascular and background pixels that are judged as a background in the segmentation result, respectively.

Figure 8 shows the comparisons of accuracy and sensitivity between the traditional Frangi filter and the proposed method on the test set. The proposed method is superior to the traditional Frangi filter in terms of the segmentation effect of most fundus retinal images. The two images in the proposed method have lesser sensitivity but significantly higher sensitivity on the remaining images compared with those in the traditional Frangi filter. Moreover, accuracy is increased while significantly improving sensitivity.

For a better assessment, the proposed method was compared with other relatively new algorithms in terms of accuracy, sensitivity, and specificity. Performance comparison of the proposed method with some of the existing methods on both the DRIVE and STARE data sets was also conducted, as shown in Tables 2 and 3.

From the performance comparison of the methods in Tables 2 and 3, the method proposed by Budak et al. [36] has the highest accuracy in the DRIVE and STARE data sets, respectively, 0.9685 and 0.9735, which are higher than the proposed method's 0.0131 and 0.0243, respectively. The method proposed by Guo et al. [35] has the highest sensitivity, respectively, 0.9589 and 0.9861, which are much higher than all other methods, but this method tends to make the specificity very low, only 0.7046 and 0.5628, respectively.

Fu et al. [34], Guo et al. [35], Budak et al. [36], and Guo et al. [37] are all based on deep learning methods for blood vessel segmentation. The disadvantage is that a large amount of data is required for learning. For medical images such as the fundus retina, obtaining enough fundus retina images is itself a challenging problem. The amount of data in the existing fundus image database is also very small, and there are large differences between different data sets. The proposed method is the same as the methods proposed by Chaudhuri et al. [6], Li et al. [7], and Barkana et al. [32]. It only uses image features and attributes to process. Compared with the methods of Chaudhuri et al. [6], the proposed method has the highest accuracy in the DRIVE data set, and the method is simple and easy to implement. Under the condition of ensuring the sensitivity, the overall accuracy is high, and the balance of the three indicators is ensured.

Vessel segmentation of fine blood vessels for fundus retinal images is difficult. Compared with other classical methods, the proposed method achieves higher accuracy because it can segment fine blood vessels well while protecting the integrity of the trunk after segmentation. Using the improved Frangi Hessian model in enhancing blood vessels not only extracts vascular feature maps under multiscale but also enhances fine branches of blood vessels effectively. In addition, the proposed method eliminates noise interferences surrounding fine blood vessels through the improved mathematical morphological operation. Hence, the proposed method highlights fine blood vessels, thus enabling accurate segmentation.

## 4. Conclusions

A blood vessel segmentation algorithm of fundus retinal images on the basis of the improved Frangi and mathematical morphology is proposed in this study. The proposed method uses the improved Frangi Hessian model to enhance blood vessels, thereby achieving the extraction of blood vessel feature maps under multiscale conditions and enhancing small blood vessels. Moreover, an improved mathematical morphological operation is used to eliminate noise interferences surrounding the fine blood vessels, considering the diameter and direction of blood vessels. Hence, fine blood vessels can be recognized as blood vessel pixels accurately in the final Otsu segmentation. The proposed method is tested by the public DRIVE and STARE data sets. According to the test results, the average segmentation accuracy, sensitivity, and specificity of retinal images in DRIVE and STARE are 95.54%, 69.42%, and 98.02% and 94.92%, 70.19%, and 97.71%, respectively. Moreover, the proposed method can maintain relatively high segmentation accuracy under the premise of ensuring segmentation sensitivity and shows good overall performances. However, the optic disk may interfere, thus influencing the segmentation effect. Hence, future studies may focus on eliminating such influences on the segmentation effect.

## Figures and Tables

**Figure 1:** Images of R, G, and B channels: (a) R channel; (b) G channel; (c) B channel.

**Figure 2:** Contrast enhancement images: (a) Enhancement by histogram equalization; (b) enhancement by CLAHE.

**Figure 3:** Multiscale vessel enhanced images: (a) Frangi filter enhancement; (b) improved Frangi filter enhancement.

**Figure 4:** Mathematical morphology processing: (a) traditional mathematical morphology; (b) subregion magnification of (a); (c) improved mathematical morphology; (d) subregion magnification of (c).

**Figure 5:** The comparison of blood vessel segmentation effect of fundus retinal image. (a) Original color fundus retinal images; (b) results of manual segmentation by the first expert; (c) results of manual segmentation by the second expert; (d) results processed by traditional Frangi filter; (e) results processed by the proposed method.

**Figure 6:** 1D cross sections of the middle row of marked subarea in the first image in Figure 5.

**Figure 7:** Detailed comparison of segmentation results. (a) Segmentation results of the proposed method; (b)~(d) are the enlarged maps of the marked detail area of the results of expert manual segmentation, traditional Frangi filter processing, and the proposed method segmentation, respectively.

**Figure 8:** Comparisons of evaluation indicators between traditional Frangi filter and the proposed method.

**Table 1:** The calculation formulas of blood vessel segmentation evaluation indicators in fundus retinal image.

Evaluation indicators	Calculation formulas
Accuracy (Acc)	Acc = (TP + TN)/(TP + FP + TN + FN)
Sensitivity (Se)	Se = TP/(TP + FN)
Specificity (Sp)	Sp = TN/(TN + FP)

**Table 2:** Performance comparison of blood vessel segmentation methods with the DRIVE data set.

Methods	Evaluation indicators		
	Acc	Se	Sp
Chaudhuri et al. [6]	0.8773	0.3357	0.9794
Li et al. [7]	0.9343	0.7154	0.9716
Barkana et al. [32]	0.9502	0.7224	0.9840
Hassanien et al. [33]	0.9388	0.7210	0.9710
Rezaee et al. [18]	0.9463	0.7189	0.9793
Zhao et al. [17]	0.9477	0.7354	0.9789
Fu et al. [34]	0.9470	0.7294	—
Guo et al. [35]	0.9613	0.9859	0.7046
Budak et al. [36]	0.9685	0.7439	0.9900
Guo et al. [37]	0.9075	0.8990	0.9283
The proposed method	0.9554	0.6942	0.9802

**Table 3:** Performance comparison of blood vessel segmentation methods with the STARE data set.

Methods	Evaluation indicators		
	Acc	Se	Sp
Li et al. [7]	0.9407	0.7192	0.9692
Barkana et al. [32]	0.9553	0.7014	0.9846
Hassanien et al. [33]	0.9468	0.6490	0.9820
Rezaee et al. [18]	0.9521	0.7202	0.9741
Zhao et al. [17]	0.9509	0.7187	0.9767
Fu et al. [34]	0.9545	0.7140	—
Guo et al. [35]	0.9539	0.9861	0.5628
Budak et al. [36]	0.9735	0.8196	0.9871
The proposed method	0.9492	0.7019	0.9771

## Data Availability

In this study, the proposed algorithm was tested on the test set of public fundus retinal images by the DRIVE database.
